The article "A rare case of chikungunya encephalitis and its management: A case report and literature review" was retracted in 2026. Reasons: fabricated or falsified data; plagiarized data; plagiarized images; overlap with other authors' work.

# A rare case of chikungunya encephalitis and its management: A case report and literature review

**DOI:** 10.1002/ccr3.8656

**Published:** 2024-03-11

**Authors:** Pugazhendi Inban, Sai Harini Chandrasekaran, Preeti Kumari Yadav, Roshini Vijayakumar, Zenia Elavia, Mansi Singh

**Affiliations:** ^1^ Department of Medicine Government Medical College Omandurar Chennai India; ^2^ Department of Medicine Cama and Albless Hospital Mumbai India; ^3^ Department of Medicine Nnamdi Azikiwe University Awka Nigeria; ^4^ Department of Medicine Bogomolets National Medical University Kyiv Ukraine

**Keywords:** cerebrospinal fluid, chikungunya virus, chikungunya virus RNA, Glasgow Coma Scale, intravenous immunoglobulin, magnetic resonance imaging

## Abstract

**Key Clinical Message:**

Chikungunya encephalitis, though rare, warrants clinical attention due to its severe complications. Early identification and appropriate management are crucial for improved outcomes in patients with this rare manifestation of chikungunya virus (CHIKV) infection.

**Abstract:**

CHIKV infection is commonly associated with fever and joint pains, but neurological complications such as encephalitis are rare. Here, we present a unique case of confirmed chikungunya encephalitis in a 12‐year‐old male exhibiting atypical neurological symptoms. The diagnostic journey involved comprehensive neuroimaging and serological investigations, revealing intriguing findings on magnetic resonance imaging and positive CHIKV RNA in serum and cerebrospinal fluid. We discuss the clinical presentation, radiological characteristics, and management strategies, emphasizing the importance of recognizing this uncommon neurological manifestation of CHIKV infection.

## 1 INTRODUCTION

Chikungunya virus (CHIKV) is an alphavirus of the family Togaviridae,^1^ with outbreaks occurring across Africa, Asia, parts of Europe, and South and Central America.^2^ The primary vectors responsible for transmitting the CHIKV are Aedes mosquitoes, particularly *Aedes aegypti* and *Aedes albopictus*. These mosquitoes are commonly found in tropical and subtropical regions.^3^ Studies have suggested that the CHIKV can be detected in the placenta, amniotic fluid, and breast milk, indicating the potential for mother‐to‐child transmission.^4^ While vertical transmission is possible, it is generally considered less common than transmission through mosquito bites.

CHIKV infection is primarily known for causing fever, headache, maculopapular rash, conjunctivitis, and arthralgia.^1^, ^5^ However, neurological complications, particularly chikungunya encephalitis, are exceedingly rare and poorly understood. Alphaviruses have been associated with viral encephalitis, leading to prolonged neurological consequences such as cognitive impairments, confusion, mood alterations, and memory decline.^6^ A study monitoring individuals infected with the alphaviruses Madariaga virus, Venezuelan equine encephalitis, and Una virus revealed persistent effects, including depression, insomnia, and dizziness, in the long term.^6^, ^7^

We report a case of chikungunya encephalitis in an elderly patient, highlighting the diagnostic challenges and management strategies.

The article "A rare case of chikungunya encephalitis and its management: A case report and literature review" was retracted in 2026. Reasons: fabricated or falsified data; plagiarized data; plagiarized images; overlap with other authors' work.

## 2 CASE PRESENTATION

### 2.1 Patient information

A 12‐year‐old male was admitted to our facility with a chief complaint of fever and joint pains persisting for 2 days, followed by a progressive decline in consciousness over the subsequent 4 days.

### 2.2 History of the present illness

The patient initially presented with a high‐grade fever and severe joint pains involving multiple joints, predominantly the wrists, knees, and ankles. Despite conservative management with antipyretics and analgesics, the fever persisted, and the joint pains intensified. Subsequently, he experienced a gradual onset of confusion and altered sensorium, prompting hospital admission.

The patient has a history of seasonal allergies and mild asthma, managed with as‐needed bronchodilators and antihistamines. He occasionally takes acetaminophen for joint pains and reports no substance abuse or tobacco use. Engaging in outdoor activities during the evenings increases his exposure to mosquitoes, aligning with the ongoing tropical season and potentially raising the risk of vector‐borne infections.

### 2.3 Physical examination

Upon admission, the patient presented as lethargic and disoriented. Vital signs showed a temperature of 38.7°C (101.7 °F), with blood pressure within normal limits, a pulse rate of 92 beats per minute, and a respiratory rate of 18 breaths per minute. During the neurological examination, an altered level of consciousness was observed, as indicated by a Glasgow Coma Scale score of 12 (E3V3M6). Reflexes and muscle strength were found to be normal, and no focal neurological deficits were evident.

Musculoskeletal examination demonstrated tenderness and swelling in multiple joints, particularly the wrists, knees, and ankles. There were no overt signs of erythema or joint effusion. A skin examination revealed no rash or palpable lesions. Cardiovascular and respiratory examinations were unremarkable.

### 2.4 Investigations and imaging

Considering the patient's deteriorating neurological status and the ongoing tropical (mosquito) season in our region, an extensive diagnostic workup was initiated. Initial laboratory investigations revealed leukopenia and thrombocytopenia, as shown in Table 1.

The article "A rare case of chikungunya encephalitis and its management: A case report and literature review" was retracted in 2026. Reasons: fabricated or falsified data; plagiarized data; plagiarized images; overlap with other authors' work.

**TABLE 1:** Complete blood count parameters, erythrocyte sedimentation rate, and C‐reactive protein values.

Lab test	Day of admission	Day 4	Day of discharge	One‐month follow‐up	Reference value
Hemoglobin	13.2 g/dL	12.8 g/dL	13.5 g/dL	13.7 g/dL	12.0–15.5 g/dL
Hematocrit	39%	38%	40%	41%	36%–46%
White blood cell count	3.6 × 10^3^/μL	5.0 × 10^3^/μL	6.2 × 10^3^/μL	7.0 × 10^3^/μL	4.0–11.0 × 10^3^/μL
Neutrophil count	5.5 × 10^3^/μL	6.2 × 10^3^/μL	5.0 × 10^3^/μL	4.8 × 10^3^/μL	2.0–7.5 × 10^3^/μL
Lymphocyte count	2.8 × 10^3^/μL	2.0 × 10^3^/μL	3.5 × 10^3^/μL	3.2 × 10^3^/μL	1.0–4.0 × 10^3^/μL
Platelet count	110 × 10^3^/μL	150 × 10^3^/μL	180 × 10^3^/μL	220 × 10^3^/μL	150–400 × 10^3^/μL
Erythrocyte sedimentation rate	15 mm/h	5 mm/h	3 mm/h	2 mm/h	0–20 mm/h
C‐reactive protein	2.1 mg/L	0.8 mg/L	0.5 mg/L	0.3 mg/L	0–3.0 mg/L
Chikungunya virus RNA (serum)	Positive	Negative	Negative	Negative	N/A
Chikungunya virus RNA (cerebrospinal fluid)	Positive	Negative	Negative	Negative	N/A

Cerebrospinal fluid (CSF) analysis displayed lymphocytic pleocytosis with an elevated protein level (details provided in Table 2).

**TABLE 2:** Cerebrospinal fluid analysis.

Cerebrospinal fluid investigations	Patient's value	Reference value
Protein	87 mg/dL	15–50 mg/dL
Glucose	63 mg/dL	45–100 mg/dL
Total white blood cells	112/cmm (100% lymphocytes)	<08/cmm

The neuroimaging studies, particularly magnetic resonance imaging (MRI) with gadolinium contrast, exhibited intriguing findings on diffusion‐weighted imaging (DWI), as shown in Figure 1, and apparent diffusion coefficient sequences. Scattered bilateral white matter lesions with periventricular diffusion‐restricted spots were observed. Notably, there was no involvement in the posterior fossa, cortical, or deep gray matter. Additionally, T2, Flair, and susceptibility‐weighted imaging in Figure 2 scans did not demonstrate significant abnormalities.

**FIGURE 1:** Magnetic resonance imaging with gadolinium contrast.

**FIGURE 2:** T2, Flair, and susceptibility‐weighted imaging.

### 2.5 Serological investigations

Serum and CSF samples were obtained for specific testing. Reverse transcription‐polymerase chain reaction for CHIKV RNA was performed. Surprisingly, both serum and CSF samples returned positive for CHIKV RNA, confirming chikungunya encephalitis serologically.

### 2.6 Diagnosis

The patient was diagnosed with a rare case of chikungunya encephalitis, supported by clinical presentation, neuroimaging findings, and positive serological confirmation of CHIKV RNA in both serum and CSF as shown in Table 1.

### 2.7 Management and follow‐up

The patient underwent intravenous immunoglobulin (IVIG) therapy for approximately 7 days, receiving a dosage of 10 mg/kg every 8 h. During the 1‐month follow‐up period, there was a noticeable improvement in neurological symptoms, marked by the resolution of confusion and joint pains. Follow‐up laboratory tests indicated a gradual normalization of complete blood count parameters, including leukopenia and thrombocytopenia. Additionally, there was a decline in inflammatory markers such as erythrocyte sedimentation rate and C‐reactive protein levels, signifying a positive response to treatment, as demonstrated in Table 1. Neuroimaging studies conducted at the follow‐up revealed a significant reduction in white matter lesions, indicating an ongoing recovery process. The overall clinical progress of the patient was highly encouraging, and with continued supportive care, a complete recovery from chikungunya encephalitis is anticipated.

The article "A rare case of chikungunya encephalitis and its management: A case report and literature review" was retracted in 2026. Reasons: fabricated or falsified data; plagiarized data; plagiarized images; overlap with other authors' work.

## 3 DISCUSSION

Chikungunya is predominantly transmitted by Aedes mosquitoes, and these mosquitoes' geographic distribution is continually expanding on a global scale. Given the absence of a known cure or vaccine for CHIKV, medical professionals worldwide must be well‐informed about the clinical aspects of CHIKV, especially considering the rising risk of the disease.^8^

CHIKV infection is primarily identified for inducing symptoms such as fever, headache, maculopapular rash, conjunctivitis, and arthralgia. However, rarely it can also cause encephalitis. The first report of neurological disease after CHIKV infection emerged during an outbreak in 1964 in Madras, India.^9^ Subsequently, neurological symptoms have been documented across various regions, including the Indian Ocean, South Asia, the Pacific islands, Southern Europe, the Caribbean, and South America.^10^ These manifestations vary from mild behavioral issues to severe acute syndromes affecting both the central nervous system and peripheral nervous system Figure 3.

**FIGURE 3:** Countries/territories with reported chikungunya cases.^10^

In this case report the diagnosis was established through the positive correlation of clinical symptoms, serological findings, CSF analysis, and neuroimaging characteristics.

Brain MRI revealed bilateral numerous small punctate lesions in the white matter with periventricular diffusion‐restricted spots. He heightened signals on DWI which is a characteristic feature observed in the early stages of chikungunya encephalitis.^11^, ^12^, ^13^ The distinctive neuroimaging findings, characterized by bilateral white matter lesions with restricted diffusion, result from cytotoxic edema attributed to plasma leakage from capillaries and venules.

Additionally, the serum and CSF samples obtained from the patient came back positive for CHIKV.

The article "A rare case of chikungunya encephalitis and its management: A case report and literature review" was retracted in 2026. Reasons: fabricated or falsified data; plagiarized data; plagiarized images; overlap with other authors' work.

In experimental investigations, both RNA and the virus itself have been identified in CSF, indicating direct neuroinvasion.^14^ However, postmortem examinations of the brain, along with histopathologic analyses, failed to identify CHIKV.^13^ Therefore, the target cell of CHIKV is still unknown.

Chikungunya encephalitis is an exceedingly rare complication of CHIKV infection, particularly noteworthy in this case due to its confirmation via serological testing in both serum and CSF. The neuroimaging findings of scattered bilateral white matter lesions with diffusion restriction and absence of enhancement align with limited existing literature on chikungunya encephalitis.

Treatment primarily focused on IVIG, and supportive care, including hydration, antipyretics, and analgesics for fever and joint pains. Studies have shown good responses in patients who are given IVIG.^15^ Additionally, neurological monitoring and symptomatic management were instituted. Given the absence of specific antiviral therapy for chikungunya, a multidisciplinary approach involving neurologists and infectious disease specialists was adopted for holistic patient care.

## 4 CONCLUSION

Chikungunya encephalitis remains a rare neurological manifestation of CHIKV infection, posing diagnostic challenges due to its atypical presentation and limited understanding. This case emphasizes the significance of considering chikungunya in the differential diagnosis of acute encephalitis, particularly in regions endemic to the virus. Further research and awareness are warranted to enhance our understanding and management of this uncommon neurological complication.

## AUTHOR CONTRIBUTIONS

**Pugazhendi Inban:** Writing – original draft. **Sai Harini Chandrasekaran:** Writing – original draft. **Preeti Kumari Yadav:** Resources; validation. **Roshini Vijayakumar:** Conceptualization; writing – review and editing. **Zenia Elavia:** Investigation; methodology. **Mansi Singh:** Writing – review and editing.

## CONFLICT OF INTEREST STATEMENT

None.

## FUNDING INFORMATION

No Funding to Disclose.

## CONSENT

Written informed consent was obtained from the patient to publish this report in accordance with the journal's patient consent policy.

## Data Availability

The datasets analyzed during the current study are available from the corresponding author upon reasonable request. Additionally, comprehensive literature sources used for the literature review are cited appropriately within the manuscript.
